# Antimicrobial misuse in pediatric urinary tract infections: recurrences and renal scarring

This article has been retracted.

**DOI:** 10.1186/s12941-018-0279-4

**Published:** 2018-06-25

**Authors:** Jayaweera Arachchige Asela Sampath Jayaweera, Mohommed Reyes

**Affiliations:** 1 Department of Microbiology, Faculty of Medicine and Allied Sciences, Rajarata University of Sri Lanka, Saliyapura, Sri Lanka; 2 Department of Pediactrics, Faculty of Medicine and Allied Sciences, Rajarata University of Sri Lanka, Saliyapura, Sri Lanka

**Keywords:** Childhood UTI, General practitioner, Empiric antimicrobial, Emergence of resistance, Bio film, Recurrent pyelonephritis and renal scarring

## Abstract

**Background:**

In children, urinary tract infection (UTI) is one of a common bacterial infection. This study was conducted to detect the uropathogen, antimicrobial susceptibility, pathogen associated with recurrences and renal scarring in children initially taken care from general practitioners and later presented to tertiary care.

**Methods:**

Every inward UTI episode, culture and antimicrobial susceptibility was done while on past 6-month, history of infections and use of antimicrobials was collected using clinical records and demonstration of antimicrobials. Children with recurrent pyelonephritis was followed and in vitro bio film formation was assessed.

**Results:**

Frequency of UTI was significantly high among infants (p = 0.03). Last 6-month, all (220) were exposed to antimicrobials. Cefixime was the commonly prescribed antimicrobial (p = 0.02). In current UTI episode, 64.5% (142/220) of children with UTI were consulted GPs’ prior to seek treatment from tertiary care pediatric unit (p = 0.02). While on follow up child who developed UTI, found urine culture isolates were significantly shifted from *E. coli* and *K. pneumoniae* to extended spectrum of beta-lactamase (ESBL) *E. coli* and *K. pneumoniae.* Out of 208 participants, 36 of them had re-current pyelonephritis (R-PN). Renal scarring (RS) was detected in 22 out of 70 patients with pyelonephritis following dimercaptosuccinic acid scan. Following each episodes of recurrent pyelonephritis 11% of new scar formation was detected (p = 0.02). Bio film forming *E. coli* and *K. pneumoniae* was significantly associated in patients with R-PN (p = 0.04).

**Discussion:**

Medical care providers often prescribe antimicrobials without having an etiological diagnosis. While continuing exposure of third generation cephalosporin and carbapenem leads to development of ESBL and CRE microbes in great. The empiric uses of antimicrobials need to be stream lined with local epidemiology and antimicrobial susceptibility pattern. R-PN in childhood leads to RS. In great, bio film formation act as the focus for such recurrences.

## Background

Urinary tract infection (UTI) is one of a common bacterial infection in children in world. It is much common among neonates and infants [1, 2]. In infants, is common among boys, thereafter the incidence is substantially rises in girls [3, 4]. Global estimated incidence of UTI among girls is 3–5%, while among boys it is 1% [5].

Since clinical features of UTI in children less than 2 years are vague, it is not generally reported as a cause of childhood morbidity [6]. The prominent risk associated with recurrent pyelonephritis in children is the tendency to develop renal scarring and progressive renal failure [7]. Permanent renal scarring has been observed after UTI in 15–60% of affected children [8]. To minimize such insult the early diagnosis and targeted antimicrobial therapy is crucial [9]. To arrive at a microbiological diagnosis, Royal college of physicians (United Kingdom) guideline stated that clean catch urine in an infant or a mid-stream urine specimen in an older child is the ideal for urine culture [10]. With conventional microbial culture antimicrobial susceptibility can be obtained in 48–72  h [11]. Therefore, in the majority of UTI cases, the treatment decision is empirical, [12] being influenced by available data reflecting antibiotic susceptibility. In the developing world where lacking local epidemiology data, choice of antimicrobials is dependent upon clinical status and clinicians experience.

Current in globe, emergences of multi drug resistance superbugs associated UTI is a common problem and it warrants use of costly antimicrobials. Extended spectrum of beta lactamases (ESBL) [13], carbapenem resistance enterobacteriaceae (CRE) [14], methicillin resistance *Staphylococcus aureus* (MRSA) [15], and vancomycin resistance enterococci (VRE) [16] are some of common superbugs. Hence, antimicrobial pipeline is dried, to curtail superbugs the use of last resorts of antimicrobials are underway.

Sri Lanka is comprised with organized public health care system and well spreaded general practitioner (GP) network. With the vigilance of parents’ care towards their child, they tend to seek care from medical practitioner in early following development of sign and symptoms. Due to paucity of validated data on empiric use of antimicrobials in childhood UTI, GPs tend to prescribed medications without proven culture evidences. With this practice, often child’s current episode would be subsided but emergence of multidrug resistance is inevitable.

Some instances with over vigilance, parents seek medications from multiple GPs. The intentions are clear as aim is to get cured. But, this act more often lead to detrimental effects as child may have ended up in inward medical care with worsening the condition. The factors contributed towards lack of response from GP and inward care would be, child having inherent or acquired uro-genital structural anomalies, physiological derangements and acquiring multidrug resistance microbes [10]. To overcome this hurdle GPs, as the first come practitioners need to pay attention in great deal. They impact can specifically pay attention towards rational use of antimicrobials [11, 12].

The data regarding the isolation frequency and antimicrobial susceptibility patterns of endemic uropathogens are less available in Sri Lanka. The aim of the present study was to determine the uropathogen isolation frequency, antimicrobial susceptibility pattern, responsible agents for recurrences and renal scarring among children subjected to seek initial medical care from GPs and presented to further care in at Teaching hospital Anuradhapura (THA), Sri Lanka.

## Methods

### Study design

This follow up study was conducted in pediatric unit, Teaching Hospital Anuradhapura, Sri Lanka from January 2013–January 2015. Six-month period from January 2013–June 2013 children having UTI was included and follow up was done for 18 months.

### Inclusion and exclusion criteria

During the study period, children up to 12 years of age admitted to pediatric ward with a clinical diagnosis of UTI were included. Since signs and symptoms of UTI and pyelonephritis vary with the age of the patient: neonates who are having fever ± and vomiting, poor feeding, jaundice and failure to thrive or part of evaluation of neonatal sepsis; infants and young children 2 months to 2 years who are having nonspecific symptoms of fever lasting longer than 48 h, as well as with poor feeding, vomiting, and diarrhea was included. Further in preschoolers and school-age children present with fever for greater than 48 h were included. Also, those who complain of abdominal pain or flank pain were included [3, 4]. Based on revised American academy of physicians (AAP) guideline on UTI in febrile infants and young children diagnosis of UTI was made by unit pediatricians [17]. Who had previous known history of antimicrobial therapy for current episode of UTI prior to attending the hospital was also included. Further, having outpatient urine culture finding concluding significant bacteriuria and from samples which grew more than one type of organism were also included.

Demographic data, complete history of current UTI episode, including the use of antibiotics from outpatient care from GPs and public health care system (inward care) and history of infectious diseases on past 6 months was gathered using clinical records and demonstration of antimicrobials. Once in every 2-month child current clinical condition and development of infectious diseases was assessed using telephone interviews. Child was followed up for 18 months to assess the development of infectious diseases including UTI while asking them to admit to pediatric unit, Teaching Hospital Anuradhapura to provide primary care.

### Clinical case definitions

Pyelonephritis is the inflammation of both the lining of the renal pelvis and the parenchyma of the kidney especially due to bacterial infection [18]. Compared to adults in children sign and symptoms are vague thus ultra sound scan of kidneys would aid the diagnosis in great. Recurrent urinary tract infection refers to ≥ 2 infections in 6 months or ≥ 3 infections in 1 year [19]. Renal scarring is a general term to describe scarring of the kidneys’ tiny blood vessels, the glomeruli, the functional units in the kidney that filter urine from the blood [7].

### Laboratory methods

In current episode urine culture was done in non-toilet trained children using clean catched urine samples following demonstration of the procedure to the guardian. In male, glans penis and foreskin while in female perineum including labia minora and majora was cleaned using antiseptics prior to obtaining the clean catch urine. From elderly children, following a video demonstration and with the aid of parent/guardian the clean catched mid-stream urine was collected to sterile containers. Semi-quantitatively by inoculating 0.001 ml of the specimen (by using a calibrated wire loop) onto the cystine lactose electrolyte deficient (CLED) agar for the isolation and identification of significant uropathogens [20, 21]. The inoculated plates were incubated for 24 h at 37 °C in aerobic and anaerobic atmosphere. Growth of a single organism with a count of ≥ 10^5^ colony-forming units (CFU)/ml were considered to represent the infection and were identified using appropriate routine identification methods including colony morphology, Gram-stain, and an in-house set of biochemical tests and further confirmed using Rapid 20 E (Enterobacteriaceae), NE (Non Enterobacteriaceae) and S (*Staphylococcus*) semi-automated identification system. Colony count was obtained using colony counter and expressed as CFU/ml.

Following each episode of pyelonephritis 2 urine cultures were done to assess the bacterial clearance. Majority of cases it was performed on day 3 and 5 while in some patients depend on C reactive protein (< 5 mg/dl-normal) and clinical response clearance culture was performed on day 5 and 7 as well [22, 23].

Further, in all children with clinically suspected pyelonephritis (fever and any of specific urinary or non-specific sign and symptoms) ultrasonography and dimercaptosuccinic acid (DMSA) [24] scan was performed to assess the renal status including renal scarring. Further, in each episodes of pyelonephritis sequentially DMSA was performed to assess the progress of renal scarring. Micturating cystourethrogram (MCUG) [25] was performed in children with pyelonephritis and recurrent UTI to detect vesicoureteral reflux (VUR).

### Bio-film formation

In-vitro bio film formation was assess using 1% percent crystal violet staining applied to polystyrene microtiter plates at 72 h and measured the optical density (OD) values [26]. This method had been validated to measure biofilm formation against laser scanning microscopy and scanning electron microscopy.

### Antimicrobial susceptibility tests

The antimicrobial susceptibility testing was performed by the disc diffusion test based on Clinical and Laboratory Standards Institute (CLSI) guidelines [27]. The following antimicrobial agents were tested: amikacin (30 μg), aztreonam (30 μg), cefepime (30 μg), cefotaxime (30 μg), cefotetan (30 μg), ceftazidime (30 μg), cefuroxime (30 μg), ceftriaxone (30 μg), cephalothin (30 μg), ciprofloxacin (5 μg), gentamicin (10 μg), meropenem (10 μg), imipenem (10 μg), piperacillin–tazobactam (100/10 μg), and tobramycin (10 μg).

### Screening and confirmatory tests for ESBL-producing strains

ESBL production confirmatory tests with ceftazidime and cefotaxime were performed by the double-disc synergy test, according to CLSI guidelines [27]. A minimum of 5-mm increase in the zone of diameter of third generation cephalosporin, tested in combination with clavulanic acid versus its zone when tested alone was accepted as an indication of extended spectrum of beta-lactamase (ESBL) production [28].

### Screening and confirmatory tests for Carbapenamases

Carbapenemase production by the *E. coli* and *K. pneumoniae* isolate was assessed using the biochemical Carba NP test [15]. The results of the Carba NP test II (which indicates the type of carbapenemase) [29], and of an MBL Etest (bioMérieux), suggested presence of metallo-β-lactamase.

### Statistical analysis

The data were double checked and transported to SAS 9.1 (2005 New Jersey.) [30]. Continuous data were presented as mean and standard deviation (SD) thus data were determined to be normally distributed and median or interquartile range (IQR) used for nonparametric data. The Chi square test or Fisher’s exact test was used to compare categorical variables and the Mann–Whitney *U* test or Kruskal–Wallis test was used to assess differences in continuous variables. The 2-way ANOVA and mean separation was performed to assess the association among parameters. Spearman correlation coefficient was used to assess the correlation between parameters. All *p*-values were two-tailed and p < 0.05 were considered statistically significant.

## Results

### Patient demographics

Two hundred and twenty children with UTI were participated and their demography and clinical presentation is displayed in Table 1. Childhood inward UTI incidence was 73.3% while acute pyelonephritis incidence was 23.3%. Recurrent pyelonephritis incidence was 11.3 per 100,000-person years. When considering age, 110 were in 1–≤ 12 months, 57 were ≥ 12–60 months and 53 were in ≥ 60 months to 12 years. Considering gender in ≥ 60 months to 12-year category male predominance was observed and other age categories showed that females were more prone to develop UTI (p = 0.02). Fever was the significant clinical presentation in study cohort (p = 0.02).

**Table 1:** Demography and clinical presentation data in study cohort

Parameter	Frequency % (n = 220)	Comments and p value
Age		
1– ≤ 12 months	50% (n = 110)	Occurrence of UTI is significantly high among infants (p = 0.03)
≥ 12–60 months	26% (n = 57)	
≥ 60 months–12 years	24% (n = 53)	
Sex male: female in;		
1–≤ 12 months	40:60	After 5 years of age male predominance was observed (p = 0.03)
≥ 12–60 months	42:58	
≥ 60 months–12 years	54:46	
Ethnicity		
Sinhala	65%	
Sri Lankan Moor	26%	
Sri Lankan Tamil	8%	
Other	1%	
Clinical presentation-prominent		
Excessive crying	7%	The most prominent clinical presentation/s were given and overlapping of symptoms were observed Fever was the commonest clinical presentations (p = 0.4)
Fever	68%	
Vomiting	36%	
Crying during micturition	28%	
Crying prior to micturition	24%	
Crying after micturition	27%	
Hematuria	22%	
Dysuria	32%	
Frequency	32%	
Loin pain	26%	
Supra-pubic pain	23%	
Drowsy	4%	

### Past 6 months

About past 6 months: infections; use of antimicrobials and current episode: treatment and inward investigation profile was displayed in Table 2. When considering clinical history and antimicrobial exposure in 6 months prior to current UTI episode, UTI (p = 0.03) and acute respiratory tract infection (p = 0.03) was significantly common in 1–≤ 12-month category while in ≥ 60 months to 12-year age category accidental wounds were significantly common (p = 0.02). Almost all were exposed to antimicrobials in last 6 months. Cefixime and co-amoxiclav was the commonly prescribed antimicrobials. Significantly less number of urine culture was done in suspected children with UTI (p = 0.02) and empirically antimicrobial was prescribed.

**Table 2:** Detail of past infections in period of 6 months, use of antimicrobials, about the current episode including treatment and inward investigation profile and follow up for next 18 months in patients with UTI

Parameter	Frequency (%) in age categories (n = 220)			p value
	1–≤ 12 months n = 110 (%)	≥ 12–60 months n = 57 (%)	≥ 60 months–12 years n = 53 (%)	
Past clinical history (6 months)-conditions to seek antimicrobial medications				
UTI	56 (50.1)	34 (59.6)	24 (45.1)	p = 0.03
ARTI	66 (0.6)	45 (78.9)	30 (56.6)	p = 0.03
AGE	32 (29.1)	14 (24.6)	14 (26.4)	–
Infection in CNS	4 (3.6)	6 (10.5)	12 (22.6)	–
IE	–	1 (1.7)	2 (3.7)	–
Abscess	12 (10.9)	10 (17.5)	12 (22.6)	–
Accidental wounds	3 (2.7)	12 (21)	23 (43.3)	p = 0.02
Use of antimicrobials	100%	100%	100%	–
ICU admissions	3 (2.7)	3 (5.2)	4 (7.5)	–
Commonly used antimicrobials in last 6 months				
Beta-lactams				
Penicillin	4 (7.2)	8 (21)	3	–
Cephalosporin	43	31	30	p = 0.02
Cefuroxime	4	5	3	–
Ceftriaxone	9	4	4	–
Cefotaxime	7	2	5	–
Cefixime	23	20	18	p = 0.02
Meropenem	8	2	4	–
Beta lactam/inhibitor	22	9	4	–
Quinolones	12	5	3	–
Macrolides	15	2	5	–
Urinary anti-septic	4	–	–	–
Glycopeptides	2	–	4	–
Current episode				
Duration of illness prior to seek care (hours ± SD)	8 ± 4	12 ± 3	22 ± 6	p < 0.05
Mode of initial treatment consultation of				
GP—local medical practitioner	23	24	24	
Consultant pediatrician	45	11	21	p < 0.05
Empirical antimicrobial prescription rate (%)	100%	100%	100%	–
UFR done (n)	34	24	26	–
Urine culture done (n)	22	12	12	–
Culture positive (n)	16	9	8	–
Duration of treatment (hours ± SD)	18 ± 4 h	20 ± 3 h	25 ± 8 h	–
Inward care				
Period taken to inward care following GP care	20 ± 4.4 h	22 ± 4.6 h	28 ± 4 h	–
Inward Urine culture done	100%	100%	100%	–
Inward Urine culture positivity (%)	31.4%	36.8%	32.2%	–
Change of prescribed antimicrobials				
Escalation	80%	88%	92%	p = 0.02
De-escalation	16%	6%	4%	–
Not changed	4%	6%	4%	–
Out come				
Hospital stay (mean days ± SD)	3 ± 1	3.5 ± 0.5	4 ± 0.8	–
Complications				
Septicemia	5	3	5	–
Renal abscess	4	4	4	–
Infective endocarditis	2	4	4	–
USS-abdomen				
Normal	90	50	44	p = 0.02
Pyelonephritis	16	5	6	
Structural anomalies				
Scaring	2	2	3	–
Follow up detail in next 18-month period				
Frequency of UTI per year	1.5 ± 1	1 ± 1	2 ± 1	–
Compliance rate of antimicrobial use				
First day	100%	100%	100%	–
Completion of dosage	60 ± 10%	50 ± 10%	52 ± 10%	–
Average cost for antimicrobials (LKR)				
1st episode	88 ± 12	112 ± 20	132 ± 54	–
Total in last 24 months	1200 ± 300	1300 ± 280	1660 ± 290	–

*UTI* urinary tract infections, *ARTI* acute respiratory tract infection, *AGE* acute gastro enteritis; Infection in *CNS* central nervous system infections, *IE* infective endocarditis, *ICU* intensive care unit

### Current UTI episode

Hundred and forty two out of 220 children with UTI were consulted a GP/pediatrician prior to seek medication from tertiary care pediatric unit (p = 0.03). Forty-eight were transferred patients from draining area including local government treatment units in the district and the province. Four children were admitted from inward private medical hospital care whiles 26 were from direct admissions who primarily seek medical care from the THA.

### GP care

Current episode of UTI compared to ≥ 60 months to 12-year category, in age 1–≤ 12 months and ≥ 12–60-month category have consulted medical care less than 6 h following development of sign and symptoms (p = 0.02). Also, in age 1–≤ 12-month category significantly seek specialized pediatric care (p = 0.02). Further, almost all who seek GP care were exposed to antimicrobials. Commonly prescribed antimicrobials were cefixime (32%), levofloxacin (22%), co-amoxiclav (26%) and cefuroxime (17%).

### Inward care

Following inward care despite of previous culture results and empiric therapy all of were subjected to assess the infective etiology following a urine culture and antibiogram. Depends on clinical status, clinicians have decided the empiric antimicrobials. It was administered following obtaining urine and blood cultures (only suspected to having pyelonephritis). Prescribed common antimicrobials were parenteral co-amoxiclav, cefuroxime, ceftriaxone and meropenem. (Table 2).

From 220 subjects 88 (40%) were found to have culture positive UTI. Common urine culture isolates were ESBL-*E. coli*, ESBL-*K. pneumoniae*, *Enterobacter cloacae* and Methicillin resistant *Staphylococcus aureus* (MRSA). Depending on clinical status, urine and blood culture results, C-reactive protein level and differential blood count, optimization of antimicrobials were done. Escalation of antimicrobials were done in 80, 88 and 92% in 1–≤ 12 months, ≥ 12–60 month and 5–12-year age groups respectively. Antimicrobial escalation was significantly high (p = 0.02) compared to de-escalation and keeping without change of initial antimicrobials.

### Follow up

#### Antimicrobial resistance pattern

Following prescribing empiric and pre-emptive antimicrobials while in haphazard manner, urine culture results and the evolution of antimicrobial resistance in study cohort in last 2 years were displayed in Fig. 1a–d. To make it easy and organized in data analysis; available culture results were divided into 6-month intervals.

**Fig. 1:** Fractions of *E. coli* and *K. pneumoniae* positive isolates and subsequent emergence of ESBL *E. coli* and *K. pneumoniae* over 24 months in 6 month intervalsin same cohort. **a** Fraction of *E.coli* positive isolates over 24 months in 6 month intervals. **b** Fraction of *K. pneumoniae* positive isolates over 24 months in 6 month intervals. **c** Fraction of ESBL-*E.coli* positive isolates over 24 months in 6 month intervals. **d** Fraction of ESBL-*K. pneumoniae* positive isolates over 24 months in 6 month intervals

Antimicrobial susceptibility patterns of ESBL-*E. coli* and ESBL-*K. pneumoniae* as most of isolates were susceptible to carbapenams (96% for meropenem) and aminoglycoside (amikacin in 90%). Four ESBL-*E. coli* and 3 ESBL-*K. pneumoniae* isolates had intermediate resistance to meropenem. Antimicrobial susceptibility of ESBL-producing isolates was displayed in Table 3.

**Table 3:** Antibiotic Susceptibilities of ESBL-Producing isolates

Antibiotic sensitivity	ESBL	
	*Escherichia coli* n = 127 (%)	*Klebsiella pneumoniae* n (%) n = 89
Meropenem	126 (96)	86 (96.6)
Piperacillin/tazobactam	76 (59.8)	52 (58.4)
Amikacin	115 (90.5)	80 (89.5)
Gentamycin	22 (17.3)	12 (13.4)
Ciprofloxacin	8 (6.2)	6 (6.7)
Trimethoprim/sulphamethoxazole	24 (18.9)	23 (25.8)
Nitrofurantoin	38 (30)	12 (13.4)

*ESBL* Extended spectrum of beta lactamases

In addition, *Staphylococcus aureus* from 2 patients, *Enterococcus fecalis* from 3 patients, *Pseudomonas aeruginosa* from 4 patients, *Proteus mirabilis* from 12 patients, *Enterobacter cloacae* from 3 patients, *Stenotrophomonas maltophilia* from 3 patients, and *Acinetobacter baumannii*, *Serratia marcescens*, *Enterobacter aerogenes*, and *Citrobacter amalonaticus* from 2 patient each were found.

During the study period 18 of them had uro-sepsis as having blood culture and urine culture positivity with same microorganism with features of pyelonephritis. Eight were following ESBL producers (8 ESBL-*E. coli* and 4 ESBL-*K. pneumoniae*). Using MBL E test 4 (2 *E. coli* and 2 *K. pneumoniae*) Metallo ß-Lactamase were detected. Remaining were following *S. aureus* 1, 3 *E. coli* and 2 *Pseudomonas aeruginosa* patients. Further, in each episode all patients showed a bacterial clearance with clinical cure. Asymptomatic bacteriuria was not detected.

#### Renal scarring

Based on DMSA scan 26 children [11.8% out of total UTI while 37% out of pyelonephritis (n = 70)] were having renal scarring while 22 of them were detected during the study. Remaining 4 were detected earlier. Two of earlier detected subjects have developed renal scarring as a sequalae of post-pyelonephritis without having history of recurrent pyelonephritis. Remaining 2 haven’t had history of pyelonephritis. Out of 26, 4 of them were infants, 15 were from ≥ 12 to 60-month while 7 were in ≥ 60 months to 12-year age and was significantly higher among ≥ 12–60-month category (p = 0.03).

Based on MCUG, 4 (100%) of them had vesicoureteral reflux (VUR). Further, they haven’t had recurrent UTI therefore we have excluded them from the analysis.

#### UTI recurrence and renal scarring

During follow up, 36 (16.3%) children had re-current UTI (pyelonephritis 32 and cystitis 4). Six of them were in 1–≤ 12 months, 17 were in ≥ 12–60 months, 13 were in ≥ 60 months to 12 years and recurrence was significantly high among children in ≥ 12–60-month group (p = 0.02). Children with UTI recurrences 6 children (4 of them having renal scarring while 2 were not) were found to have VUR.

Patients with recurrent pyelonephritis their sequential renal DMSA scan showed significant (p = 0.02) progressive renal scarring and positive correlation with recurrences (Spearman’s correlation co-efficient 0.11). In each episode of recurrent pyelonephritis 11% renal scarring was newly developed.

#### UTI recurrences and bio-film formation

Thirty-two out of 36 children with UTI recurrences were continuously positive for same microorganism in subsequent urine cultures (22 of them having *E. coli* and 10 of them having *K. pneumoniae*). Antibiogram of sequentially detected *E. coli* and *K. pneumoniae* isolates were almost similar. Both *E. coli* and *K. pneumoniae* were detected to having beta-lactam/beta-lactam inhibitor resistance (resistance to co-amoxiclav) and was sensitive to third generation cephalosporin, quinolones and aminoglycosides. Those 32 subjects’ urine culture isolates were assessed for bio film formation. Isolates from successive final 3 UTI episodes were used to assess in vitro bio film formation.

*Escherichia coli* (n = 22) was detected in children with recurrent pyelonephritis. Sixteen (72.7%) were in children with recurrent pyelonephritis with renal scarring. Six (42.8%) *E. coli* isolates were detected in children with recurrent pyelonephritis without having renal scarring. The OD values for *E. coli* was significantly low (OD mean ± SD 0.26 ± 0.20) in the recurrent pyelonephritis without having renal scarring subjects than in recurrent pyelonephritis having renal scarring. (OD mean ± SD 0.64 ± 0.26) (p = 0.01).

*Klebsiella pneumoniae* was detected in 8 children with recurrent pyelonephritis (6 having renal scarring while 2 were without renal scarring) while 2 of them were having recurrent cystitis (no renal scarring was detected). The OD values for *K. pneumoniae* was significantly low (OD mean ± SD 0.22 ± 0.12) in children with recurrent pyelonephritis without having renal scarring than in recurrent UTI having renal scarring (OD mean ± SD 0.44 ± 0.13) (p = 0.03) (Table 4).

**Table 4:** Demography and clinical presentation of subjects having renal scarring with UTI recurrences

	Subjects with recurrent UTI (n = 36)		
	Renal scarring (n = 22)	No renal scarring (n = 14)	p value
Age at presentation (mean ± SD year)	3.5 ± 0.9	1.9 ± 0.7	> 0.05
Gender (male: female)	14:4	11:7	0.04
UTI frequency (mean ± SD per year)	3.5 ± 0.3	1.7 ± 0.5	0.04
Type of UTI			
Pyelonephritis	22 (100%)	10 (71.4%)	0.03
Other UTIs	0	4 (38.6%)	0.03
Biofilm formation in patients with pyelonephritis			
*E. coli*	16 (72.7%)	6 (42.8%)	0.04
*K. pneumoniae*	6 (27.3%)	2 (14.3%)	0.04
Vesico-ureteral reflux	4 (18.2%)	2 (19.3%)	> 0.05

p < 0.05 considered as significant

## Discussion

UTI prevalence greatly varies with gender, age, structural and functional urological anomalies. In our study, culture positive UTI incidence was 40% while a recent study in India showed incidence of culture positive UTI as 35.4% [30]. In our study based on DMSA scan, 37% was found to have renal scarring. A recent study in India shows with DMSA scan 47.8% of children was having renal scarring [31]. Renal scarring leads to acute renal parenchymal damage and subsequent permanent damage [32]. Extensive scarring may progress to further renal insult with later development of hypertension with decreased renal function, proteinuria, and end-stage renal disease [29]. Risk factors for renal scar formation in children following UTI have been reported to include: age at presentation; gender; occurrence of recurrences; high grade fever; delay in diagnosis and treatment; presence of VUR. In addition, total white blood cell count, erythrocyte sedimentation rate, and C-reactive protein (CRP) level; bacterial virulence; host defense factors; and genetic susceptibility also considered [33–37]. In most studies, significance of acute pyelonephritis, development of recurrent UTI, chronic pyelonephritis and having VUR are given as key contributory factors for development of renal scarring. In our study, 4 out of 6 children with UVR had renal scarring. Also children having VUR (6 out of 6) had recurrent UTI. But, VUR was not significantly associated with renal scar formation following recurrent pyelonephritis. A recent study in South Korea showed rate of scar formation was significantly higher in infants with VUR than in those without (39.4% vs. 7.5%) [38]. Further, the relationship between VUR and renal scar formation cannot be accurately determined in older children because VUR may improve or resolve over time. Therefore, older children without VUR at the time of investigation may have previously had VUR.

Development of acute pyelonephritis (APN) among children may leads to renal scarring. Formation of renal scarring is a result of a complex interaction between host and bacterial factors. Renal scarring can develop following acute pyelonephritis as a post-pyelonephritis sequalae. Further follow up studies on children related to chronic pyelonephritis and subsequent development of renal scarring is well described [7].

We have found that children having recurrent pyelonephritis are more prone to develop renal scarring. In our study following each episodes of recurrent pyelonephritis 11% of new scar formation was detected. A recent meta-analysis related to DMSA scintigraphy has demonstrated an average of 46% of development of renal scarring after occurrence of acute pyelonephritis, with a variation of 26–62%, depending upon the region of the world [8]. In between each acute pyelonephritis episode, ultra-sonography scan (USS) showed renal resolution while follow up urine culture on day 3 and 7 both were negative. This signifies the clinical and microbiological cure of each acute episodes. Subsequently in follow up, an individual with acute pyelonephritis episodes the urine culture became positive with similar organism. This was further confirmed by having similar antibiogram. Also, we have found that, it was significantly associated with bio film forming *E. coli* and *K. pneumoniae.*

Bacterial biofilms are associated with a large number of persistent and chronic infections. Biofilm-dwelling bacteria are particularly resistant to antibiotics and immune defenses, which makes it hard, impact impossible to eradicate biofilm-associated infections [17]. Bio film formation is quite common among implants and when medical devices kept long including urinary, other catheter and venous lines. In addition, formation of bio film over epithelia being described thus it acts as a nidus for chronic persistent or recurrent infections among healthy as well as compromised individuals [39, 40]. A European study describes the potential roll of bio film formation in development of recurrent pyelonephritis [26]. In our study, *E. coli* and *K. pneumoniae* bio film formation was significantly associated with group who was having recurrent pyelonephritis and renal scarring. Therefore, the bio film associated pyelonephritis can be a potential causative factor for development of renal scarring.

Contrary, we haven’t performed DMSA scan following clinical and microbiological resolution of each acute pyelonephritis episode. We have performed USS but its sensitivity is low thus ongoing renal insult following each pyelonephritis episode cannot be excluded. Further, in each episode the type of antimicrobial and its dosage was given based on antimicrobial susceptibility. This could lead to clinical cure or temporal suppression of impending bio-film associated bacteriuria and pyelonephritis.

The children with acute and recurrent episodes of pyelonephritis was treated according to AAP 2011 revised guidelines [41]. Adherence to treatment guidelines, use of appropriate targeted antimicrobial based on susceptibility of *E. coli* and *K. pneumoniae* isolates would lead to clinical cure and prevented the emergence of superbugs like ESBL and CRE. But all isolates from recurrent pyelonephritis were having beta lactamase inhibitor resistance. Focus of such stains could be nosocomial in origin thus all of them were had at least one episode of hospitalization prior to recruiting our study. Also, in past they were exposed to co-amoxiclav in great.

Other hand since they were having bio film, the antimicrobial penetration to the vicinity is poorer. In bio film forming bacteria, their metabolic characteristics differs from planktonic single cell strains. Therefor even with appropriate antimicrobials the cidal effect is low and it would ultimately lead to recurrences.

Further, multidrug-resistant gram-negative bacteria are a growing problem worldwide. ESBLs are plasmid-mediated groups of enzymes that hydrolyze penicillin, third generation cephalosporin, and aztreonam [42]. Carbapenems often spared thus reserved as effective first line of therapy [43]. This study signifies the most common causes of pediatric urinary tract infections are following Enterobacteriaceae such as *E. coli* and *K. pneumoniae.* Is compatible (40%) with study conducted in Southern parts of Sri Lanka in a tertiary care hospital in > 1-year age population [44]. Also, in western part of Sri Lanka in adult population having higher incidence (33%) [45]. Data on ESBL-Enterobacteriaceae incidence among pediatric population in Sri Lanka is scanty. Considering south Asian territory, it has highest incidence among all population. A recent study done in Nepal in pediatric population and it was 38.9%, [46] in Pakistan it was 50.9% [47], while in India it was 42% [48].

Further our cohort gradual rise of ESBL *E. coli* and *K. pneumoniae* was detected among UTI recurrences. Following unrestricted use of third generation cephalosporins including cefixime for pediatric UTI was high. Similarly, in Iran showed 32% of community and 42% of nosocomial isolates were having ESBL production. Further, distribution of ESBL-positive UTIs in Turkey was 3.6% in 2004, 3.9% in 2005, and 4.2% in 2006 [49]. The factors related to high and rising frequency of ESBL phenotypes are previous hospitalization, previous bacterial infection, urinary abnormalities, previous third-generation cephalosporins treatment, recurrent urinary tract infections, and presence of high-level and multi-drug resistance isolates [50].

In addition to ESBL, urinary and blood isolates of carbapenem resistance enterobacteriaceae (CRE) was detected. In Asian countries emergence of CRE cases were observed but it still remains low. A recent study in mainland China, the imipenem resistance of *E. coli* and *K. pneumonia* in 2004–2005 is 0.0 and 0.7% [51], while the rate increases to 0.5 and 2.7% in 2010 [52]. In Korea, the carbapenems resistance also follows such tendency. This could be due to lack of surveillance or could be due to under reporting. Since prudent use of antimicrobials is happening in day by day, the emergence of superbugs is inevitable but low prevalence need to be explained. In our study, all subjects with MBL *Enterobacteriaceae* sp. isolates were having closed contacts with piggery and poultry [53]. Animal husbandry is a well-known risk factor for acquisition of CRE and other superbugs.

Sri Lanka comprises well spread public as well as private medical care service. Often due to convenience and with the vigilance guardian seek medical care from the GP practice in great. More often GPs tend to prescribe antimicrobials for infective diseases without arranging investigations for detection of the etiology. In addition, in public sector clinicians tend to prescribe antimicrobials in similar manner. Often child admitted to tertiary care facility is ill and warrant an immediate therapy. Perhaps this empiric use of antimicrobials would lead to clinical cure but often this would lead to development of multi-drug resistance microbes. We have evaluated the continuous antimicrobial exposure among study population. Among them the spectrum of sensitivity has remarkably changed thus ultimately leads to development of super bugs like ESBL *E. coli* and *K. pneumoniae* strains in great. Commonly prescribed such antimicrobial was third generation cephalosporin the Cefixime. This would lead to selection of resistant flora while killing sensitive microbes in great. Other hand when these patients are having continuously exposed to antimicrobials and this would accelerate the emergence of multi drug resistant strains. Simultaneously, several hospital admissions would lead to acquisition of hospital flora where super bugs are common.

Other hand to obtained conventional culture result it may take 48–72 h. The waiting time is prolonged. Therefore, GPs reluctant to request urine culture and antimicrobial susceptibility results. Also, in resource poor settings, conducting a conventional urine culture on a regular basis is costly and cumbersome.

This study highlights the importance of arriving at an etiological diagnosis following UTI prior to commencing antimicrobials. Impact targeted therapy is gold standard. Therefor by knowing local epidemiology of UTI causing microbes and the antimicrobial susceptibility pattern will guide the clinicians to select appropriate antimicrobials. Considering the facts, the policies and practices related to current clinical practice in public and private sector in Sri Lanka is needed to be stream lined.

### Limitations of our study

As a part of this study, to assess empiric use of antimicrobials from GPs we employed a method to demonstrate different type of antimicrobial preparations in different trade names and we have asked parents/guardians to identify them. Since this was being a recalling method, the validity is questionable.

Also, instead of phenotypic identification of ESBL and CRE, we have not performed genotyping of ESBL, CRE. Also, in isolates from recurrent pyelonephritis (inhibitor resistant *E. coli* and *K. pneumoniae*) we haven’t performed genotyping and sequencing to confirm the possibility of detecting similar strain.

While analyzing the association between age and recurrences we haven’t performed a multivariable analysis to account for confounding. Limited number of patients with recurrences would be a limiting factor for such analysis. Further, in future conducting a follow up multi-centered study with large sample would be helpful to explain the possible associations.

## Conclusion

In routine, medical care providers tend to prescribe antimicrobials without having an etiological diagnosis. This malpractice need to rectify from at grass root level including general practitioners and medical undergraduates. Following haphazard manner of exposure of third generation cephalosporin specially cefixime would leads to development of ESBL microbes in great. Also, use of carbapenems leads to emergence of MBLs. Further, recurrent pyelonephritis would lead to renal scarring. Possible bio film formation would act as the focus for such recurrences. For the treatment and prevention of recurrences, possibility of bacterial bio film formation among anatomical vicinities need to concern. In addition, the UTI antimicrobial prescription guidelines need to be streamlined with the local epidemiology and infectious control practices.

In future, use of bio film formation inhibitors and development of methods for disruption of bio films will be demanding. This study would highlight the importance of rational use of antimicrobials among pediatric UTI.

## Abbreviations

UTI: urinary tract infection
GP: general practitioner
THA: Teaching Hospital Anuradhapura
CLED: cystine lactose electrolyte deficient
CLSI: Clinical and Laboratory Standards Institute
ESBL: extended spectrum of beta-lactamase
SAS: Statistical Analysis System
ESBL-*E. coli*: extended spectrum of beta-lactamase producing *Escherichia coli*
ESBL-*K. pneumoniae*: Extended spectrum of beta-lactamase producing *Klebsiella pneumoniae*
CRE: Carbapenemase resistance enterobacteriaceae
MRSA: *Methicillin resistant Staphylococcus aureus*
OD: optical density
DMSA: dimercaptosuccinic acid
MCUG: micturating cystourethrogram
VUR: vesicoureteral reflux
